RETRACTED

# Experimental and theoretical investigations of Erbium complex: DNA/BSA interaction, anticancer and antibacterial studies

**DOI:** 10.3389/fchem.2023.1266520

**Published:** 2023-08-28

**Authors:** Raid D. Thanoon, Emam Atiyah Ibadi, Irfan Ahmad, Hassan Thoulfikar A. Alamir, Marim Alwan, Furqan S. Hashim, Donia Waleed Khaled, Adnan Taan Alkhafaji, Mohammed Asiri, Ali Alsaalamy

**Affiliations:** ^1^ Department of Medical Biochemical Analysis, Cihan University-Erbil, Kurdistan Region, Iraq; ^2^ Department of Pharmacy, Al-Mustaqbal University College, Babylon, Iraq; ^3^ Department of Clinical Laboratory Sciences, College of Applied Medical Sciences, King Khalid University, Abha, Saudi Arabia; ^4^ Department of Pharmaceutics, Faculty of Pharmacy, University of Al-Ameed, Karbala, Iraq; ^5^ Medical Lab Techniques, College of Medical Technology, Al-Farahidi University, Baghdad, Iraq; ^6^ Department of Medical Laboratories Technology, Al-Nisour University College, Baghdad, Iraq; ^7^ Department of Optical Techniques, AlNoor University College, Mosul, Iraq; ^8^ Cardiology Department, College of Medicine, Al-Ayen University, Nasiriyah, Iraq; ^9^ College of Technical Engineering, Imam Ja’afar Al‐Sadiq University, Baghdad, Iraq

**Keywords:** Er complex, DNA and BSA binding, molecular docking, antimicrobial properties, anticancer properties

## Abstract

To assess the biological potential of an Er complex that contains a 2,2'-bipyridine ligand, various techniques such as multispectral and molecular modeling procedures were utilized to examine its DNA-binding ability, BSA binding affinity, antimicrobial effects, and anticancer properties. By analyzing fluorescent information and employing the vant’ Hoff equation, important parameters such as the innate docking coefficient (K_b_), Stern-Volmer coefficient (K_SV_), and thermodynamic properties including modifications in liberated energy (ΔG°), enthalpy (∆H°), and entropy (∆S°) were determined. The trial findings suggest that the compound can bind to DNA, primarily through groove binding. Additionally, the engagement between the Er compound and the protein BSA was examined using emission spectroscopy technique, revealing a powerful binding affinity between the compound and BSA. The Er complex binds to BSA primarily via hydrogen links and van der Waals forces, as indicated by the adverse values of ΔH° and ∆S°. Through a static quenching process, the complex significantly reduces the intrinsic fluorescence of BSA. Molecular binding calculations and rivalrous binding trials confirm that this compound dock to hydrophobic remains found in site III of BSA. Additionally, the Er complex demonstrates promising results in terms of its anticancer and antimicrobial activities based on screening tests.

RETRACTED

## 1 Introduction

Cancer continues to be a significant health issue in our community, and it holds a central position in the realm of medicinal chemistry at present (Mamedova et al., 2019; Tohma et al., 2019; Tugrak et al., 2019). Following the breakthrough discovery of cisplatin and its implementation in clinical therapy, scientists have dedicated significant efforts towards synthesizing a variety of platinum-based drugs (Zeng et al., 2020; Chen et al., 2023). The objective behind these endeavors is to develop alternatives that exhibit reduced toxicity to healthy tissues and can effectively combat tumors resistant to cisplatin. The primary aim in the development of non-platinum anticancer medications is to address the limitations associated with platinum drugs, such as their substantial toxicity to healthy tissues, the limited spectrum of activity, and the development of acquired resistance after treatment. Consequently, the pursuit of discovering novel non-platinum drugs with fewer side effects holds great importance within the realm of pharmaceutical chemistry (Zhang et al., 2020; Chen et al., 2021; Fu et al., 2021; Lin et al., 2021; Lou et al., 2021; Xu et al., 2021; Cong et al., 2022; Majidi et al., 2022; Zhao et al., 2023a; Zhao et al., 2023b).

Lanthanide elements have attracted significant attention in comparison to other metals due to their distinct luminescence, magnetism and crucially, their remarkable efficacy as catalysts in breaking down stable phosphodiester bonds through hydrolysis. This process generates DNA fragments that can be easily reconnected, which highlights a notable advantage of lanthanides over agents that cleave DNA through oxidation (Türkeş et al., 2019; Zhang et al., 2022b; Cao et al., 2022).

Lanthanides have garnered interest for their potential applications in oncological treatment and their use in dyes for MRI. These elements can be administered into the body, processed, and eventually discharged into the ecosystem. However, when employing lanthanides in biomedical practices, it is necessary to synthesize complex systems with specific biological activity, such as selective binding to biomolecules. In recent decades, significant research efforts have been dedicated to characterizing lanthanide compounds including 1,10-phenanthroline or 2,2′-bipyridine bindings. It has been illustrated that the inclusion of these bindings in the structure of europium compounds is crucial for enhancing their cytotoxicity (Khorasani-Motlagh et al., 2013).

Furthermore, these ligands exhibit a high absorption of UV light and efficiently transmit the energy from the bindings to the metal midpoint through an “antenna impact.” This characteristic enables primary stimulation of the lanthanide ions, which have inherently diminished absorption coefficients. Additionally, the bindings serve to safeguard the lanthanide ions from vibration linkage that could potentially suppress their luminescence (Khorasani-Motlagh et al., 2013; Lei et al., 2022; Cao et al., 2023; Tang et al., 2023).

RETRACTED

The binding of DNA is a crucial process for its functioning. To enhance the effectiveness of chemotherapeutic agents and develop improved anticancer drugs, it is necessary to investigate how metal compounds engage alongside DNA. In recent times, there have been remarkable and captivating research endeavors focusing on the connection between transition metal ions and nucleic acids due to their significance in the advancement of new tools for biotechnology and medicine. These investigations also have a vital function in comprehending the toxicity of medication that incorporates metal ions (Shahabadi et al., 2010).

The way compounds and metal compounds interact primarily relies on their organization and the characteristics of their bindings. Metal compounds can engage alongside DNA through covalent or non-covalent means, for example, intercalation, static electric interactions, or groove-binding. Additionally, they can potentially cause the separation of the DNA double helix (Pagoni et al., 2019).

Serum albumins, which are highly prevalent proteins in the plasma of mammals, play a crucial role in transporting metal ions and medication throughout the bloodstream to various cells and tissues. Among these proteins, BSA (bovine serum albumin) is extensively researched owing to its likeness in structure to human serum albumin. BSA contains two tryptophan residues located at positions 134 and 212 (Pagoni et al., 2019; Song et al., 2020).

To explore improved properties and build upon previous findings, our study focused on evaluating the bioactivities of a new compound containing Er(III) and a 2,2'-bipyridine ligand, named [Er(Bpy)_2_Cl_3_(OH_2_)]. Our goal was to investigate its potential as a novel probe for (BSA) and calf thymus DNA (CT-DNA), while also searching for new anticancer agents. The attaching interactions amidst the Erbium compound and BSA/CT-DNA were analyzed using techniques such as emission spectroscopic analysis, and viscometry. Furthermore, we examined the complex’s properties as an anticancer and antibacterial agent.

## 2 Experimental

### 2.1 Chemicals and physical measurements

We utilized chemicals of reagent grade from various suppliers without any additional purification. Sigma and Merck Companies were the sources for all other chemicals. The mononuclear complex was produced following the previously documented procedure (Aramesh-Boroujeni et al., 2018).

RETRACTED

Fluorescent spectra were obtained using a (PERKIN ELMER LS-3) apparatus, with a (1.0 cm) quartz container being used. The electronic spectra were measured utilizing an Analytic Jena SPECORD S100 spectrometer equipped with a photodiode collection probe and a thermostat cell compartment. Viscosity trials were conducted using a SCHOT AVS 450 viscosity analyzer, which was submerged in a thermostatic bath to preserve an unchanging temperature.

### 2.2 Synthesis and characterization of the Erbium complex

The Er complex was prepared by the literature method (Hussain et al., 2004). An ethanol solution of erbium chloride (5.97 × 10^−4^ mol, 100 mg) was added drop wise to the 2,2'-bipyridine (5.48 × 10^−4^ mol, 85.6 mg) dissolved in ethanol (5 mL). The resultant mixture was refluxed at 243 K for 5 hours. Then, the resulting precipitate was filtered. It was washed with ethanol and dried (yield 69%). Anal. Found (Calc.) (C_20_H_18_Cl_3_N_4_OEr): C, 39.74 (39.12); H, 2.98 (2.81); N, 9.27 (8.93). FT-IR (cm^−1^): 1,593 (C=N), 1,430–1,469 (C=C), 729–770 (C–H). ^1^H NMR (400 MHz, D_2_O): δ (ppm) 4.75 (H_2_O, broad) and 8.34, 7.69, 7.24 (H-bpy, broad). Electronic absorption (H_2_O): 232, 280 nm.

### 2.3 Preparation of stock solutions

All trials in connection with the engagement of the Er(III) compound with DNA and BSA were conducted in a buffer, Tris(hydroxymethyl)aminomethane (Tris) at a concentration of 5 mM, and sodium chloride (NaCl) at a concentration of 50 mM were used. The pH of the buffer was modified to 7.2 using hydrochloric acid. The focus point of the DNA stock solution was established by spectrophotometric measurement using the molar absorptivity value (ε) of 6600 M^−1^cm^−1^ at 260 nm. The cleanliness of the DNA was assessed by calculating the absorption level A_260_/A_280_. A value above 1.8 for A_260_/A_280_ shows that the DNA was suitably clean and devoid of protein contamination (Yu et al., 2009).

Furthermore, the amount of ethidium bromide present was determined by measuring its concentration using absorption spectroscopic analysis, presuming an extinction constant (ε) of 5450 M^−1^cm^−1^ at 480 nm. Additionally, the amount of BSA present was determined by measuring its concentration by utilizing the extinction coefficient of 44,300 M^−1^ cm^−1^ at 280 nm (Anjomshoa et al., 2014; Aramesh-Boroujeni and Jahani, 2022). All stock solutions were kept at 4 °C and utilized within 96 h of arrangement. The steadiness of the Erbium compound in an aqueous solution was evaluated by observation of its UV-Vis spectrum at different incubation hours. The widths of both the excitation and emission slits were set at 10.0 nm.

RETRACTED

### 2.4 DNA-binding studies

Fluorescence emission graphs were collected at different heat levels utilizing an excitation wave period of 280 nm and an emission wave period of 338 nm. To examine the fluorescence-suppressing productivity, various concentrations of DNA, ranging from 0.0 to 14.1 μM, were added to constant levels of the Erbium (III) compound at 1.0 µM. The fluorescence-suppressing efficiency was quantified utilizing the K_SV_, which is determined by the following equation (Calvillo-Páez et al., 2018):

$$\frac{F_{0}}{F}=1+K_{SV}\left[Q\right]$$ (1)

In the provided formula, F and F_0_ represent the fluorescence strengths of the Erbium complex in the existence and lack of the suppressor (DNA), individually. [Q] Indicates the DNA concentration. By employing Eq. 2, the docking coefficient (K_b_) and the quantity of attaching spots (n) for the DNA-Er compound framework can be estimated (Medjedović et al., 2020):

$$\log\frac{F_{0}-F}{F}={\log K}_{b}+nlog\left[Q\right]$$ (2)

Eqs 3, 4 were utilized to derive the thermodynamic parameters:

$$\ln K_{b}=-\frac{\Delta G^{0}}{RT}=-\frac{\Delta H^{0}}{R}\left(\frac{1}{T}\right)+\frac{\Delta S^{0}}{R}$$ (3)

ΔG˚=ΔH˚−TΔS˚ (4)

To examine the competitive binding between the Er-complex and EtBr, the system consisting of DNA alone and the Er-complex was excited at 525 nm. Emission experiments were conducted by gradually adding the Er-compound (ranging from 0 to 145.0 µM) to a solution consisting of 140 µM DNA and 8.0 µM EtBr.

### 2.5 BSA-binding studies

Additionally, emission titrations were conducted at various heat levels (λ_ex_ = 280, λ_em_ = 347, T = 295, 298, 300, and 303 K), with the BSA concentration held constant at 3.0 µM and the Er- complex density increasing from 0 to 6.5 µM. The quantities of K_SV_, K_b_, n, and thermochemical factors for the engagement amidst the Er- compound and BSA at the four heat levels can be calculated using Eqs 1–4, respectively. In these equations, [Q] shows the concentration of the compound.

### 2.6 Docking setup

In this research, the binding calculations were performed using Autodock4.2.2, which is considered one of the top docking packages. The BSA crystal compound (PDB ID: 3v03) and the DNA dodecamer dual (CGCGAATTCGCG)_2_ (PDB ID: 1BNA) were obtained from the Brookhaven Protein Information Center. The protein data file was prepared by removing water molecules determined by crystallography and adding any missing hydrogen atoms to the protein compounds. The 3D structure of this compound was then enhanced using the Becke-3-factor Lee-Yang-Parr (B3LYP) hybrid concentration operational concept at the 6–31 G** basis fixed level, using the ORCA quantum chemistry application (Neese, 2012). To facilitate the binding process, a grid chart with dimensions of 80 × 80 × 80 points and a spacing of 0.375 Å was created. Afterward, 200 different binding computations were performed using the Lamarckian genetic algorithm in conjunction with the nearby seek method (Morris et al., 1998). Each docking calculation involved a total of 25,000,000 energy evaluations.

RETRACTED

### 2.7 Analysis of cytotoxicity (MTT examination)

The effectiveness of the Er-compound in fighting cancer was examined through the MTT assay on A-549 and HeLa cell lines. The HeLa and MCF-7 cell lines took place in a moistened environment with 5% CO_2_ at 37°C and were exposed to varying concentrations of the Er complex for 1 day. Following this, an answer” of MTT (10 μL, 12 mM) was introduced and the plates were kept in an incubator for 4 h. The growth medium was then discarded, and DMSO (50 μL) was added to the wells, which were subsequently washed in the company of phosphate-buffered saline and incubated for 10 min. In anticancer trainings, the time was 48 h. The IC_50_, which represents the level at which 50% inhibition occurs, was computed at 545 nm using an ELISA examiner, as described by Eq. 5 (Mohamadi et al., 2017):

$$\%\text{ Cell Cytotoxicity}=\left[1-\left(\text{Drug Absorption}/\text{Control Absorption}\right)\right]\times 100$$ (5)

### 2.8 Antimicrobial activity of complex

The antibacterial potential of the complex was examined using minimum inhibitory concentration (MIC) *in vitro* (Liu et al., 2023). Various bacterial strains were selected for the study, including (*Pseudomonas aeruginosa*; *P. aeruginosa* ATCC 27853 and *Escherichia coli*; *E. coli* ATCC 25922), two Gram-positive standard strains of bacteria (*Enterococcus faecalis*; *E. faecalis* ATCC 11700 and *Staphylococcus aureus*; *S. aureus* ATCC 25923). The Mueller-Hinton agar was used as the growth average for the bacteria and was prepared in Petri plates. Next, the bacterial cultures and yeast that showed sensitivity to the complex were further examined for their (MIC) values utilizing the micro-well reduction examination procedure. Concentrations ranging from 1,024 to 2 μg/mL were tested, and the assays were conducted in DMSO. This method allowed for the quantitative determination of MIC values.

### 2.9 Statistical analysis

The data have been statistically analyzed utilizing the one-way analysis of variance (ANOVA), where *p* values < 0.05 have been considered statistically substantial. The results of three independent tests were provided as the mean ± SD.

## 3 Results and discussion

### 3.1 DNA experiments

#### 3.1.1 Fluorescence studies

Upon excitation with a wavelength of 280 nm, the Er-compound exhibited a prominent emission band at 338 nm. Figure 1 presents the emission graph of the Er-compound both in the existence and lack of DNA. As the concentration of DNA increased, a slow diminish in fluorescence strength was observed in the Er-complex, indicating that DNA suppresses the intrinsic fluorescence of the complex.

RETRACTED

**FIGURE 1:** **(A)** Emission spectra of Er-complex in the absence and existence of different DNA concentrations. **(B)** The F_0_/F vs. [DNA] plots.

Quenching can happen through various methods, typically labeled as dynamic and static suppressing. Dynamic suppressing involves the interaction amidst the fluorophore (Er-compound) and the quencher (DNA) while the transient existence of the excited condition. On the flip side, static quenching mentions the creation of a compound amidst the fluorophore and the suppressor (Er-compound-DNA). Dynamic quenching relies on diffusion, and greater heat levels, which increase the diffusion coefficients, can lead to an increase in the static quenching constant (K_SV_). However, as the heat level expands, the steadiness of the compounds may diminish, occurring in diminished values of K_SV_. The fluorescence quenching phenomenon can be explained by the Stern-Volmer formula (Eq. 1) (Shahabadi et al., 2017).

Table 1 presents the obtained values for the (K_SV_) using the equation mentioned earlier. In this study, as the heat level elevated from 295 K to 303 K, the K_SV_ reduced from 4.95 × 10^4^ M^−1^ to 5.80 × 10^4^ M^−1^ for the complex (as shown in Figure 1B; Table 1). This indicates that the suppressing procedure may be attributed to dynamic suppressing.

**TABLE 1:** The Stern-Volmer constant (K_SV_), the binding constant (K_b_), number of the binding sites (n), and thermodynamic parameters (ΔS˚, ΔH˚, and ∆G˚) for the interaction of DNA with Er-complex at various temperatures.

(K) T	K_SV_ × 10^−4^ (M^−1^)	Kb × 10^−4^ (M^−1^)	n	ΔS˚ (J/mol.K)	ΔH˚ (kJ/mol)	∆G˚ (kJ/mol)
295	7.60 ± 0.06	2.69 ± 0.05	0.92			−23.85 ± 0.04
298	7.81 ± 0.03	4.26 ± 0.07	0.95	408.63 ± 0.04	95.47 ± 0.05	−24.93 ± 0.06
301	8.95 ± 0.05	6.02 ± 0.04	0.97			−25.74 ± 0.07
303	9.35 ± 0.04	7.58 ± 0.06	0.98			−26.28 ± 0.04

The binding coefficient (K_b_) and the number of binding sites (n) for the development of the compound amidst the Er-compound and DNA were determined utilizing Eq. 2 (Figure 2A). In this research, the binding constants of the compound were measured at various heat levels and are displayed in Table 1. At room temperature, the value of K_b_ for the Er-compound was detected to be 1.66 × 10^4^ M^−1^.

RETRACTED

**FIGURE 2:** **(A)** The plot of log((F_0_-F)/F) against log([DNA]/µM) at different temperatures. **(B)** van’t Hoff plot for the interaction of Er-complex with DNA.

#### 3.1.2 Determination of thermodynamic parameters

The graph displayed in Figure 2B, showing the connection amidst natural lnK_b_ and the reciprocal of temperature (1/T), enables us to determine the values of (ΔH˚), (ΔS˚), and liberated energy (ΔG˚) changes using the van’t Hoff formula (Eqs 4, 5).

The thermodynamic properties of the compound are presented in Table 1. Based on the numerical data of enthalpy (ΔH˚) and entropy (ΔS˚), we can deduce the mode of engagement between the complex and biomolecules such as DNA. Three conclusions can be drawn: 1) When ΔH˚ > 0 and ΔS˚ > 0, the engagement is motivated by hydrophobic forces. 2) When ΔH˚ < 0 and ΔS˚ < 0, the interaction involves van der Waals forces and hydrogen bonds. 3) When ΔH˚ < 0 and ΔS˚ > 0, the interaction is governed by electrostatic interactions. Furthermore, the adverse value of ΔG˚ indicates that the procedure of DNA interaction is unprompted. Additionally, the positive values of ΔH˚ and ΔS˚ suggest that hydrophobic forces have an important function in the binding of the compound to DNA (Shahabadi et al., 2017).

#### 3.1.3 Iodide quenching studies

To earn more insights into the engagement amidst the suggested compound and DNA, the fluorescence suppressing technique was employed. The study involved measuring the fluorescence intensity during the lack and existence of DNA, with iodide ions serving as the quenching agent. Since the adversely energized phosphate backbone of DNA repels anionic quenchers, it can be inferred that small molecules bound through intercalation would be shielded in the existence of these anionic quenchers. Conversely, if the docking occurs through groove binding, the fluorescence emission would be significantly enhanced in the presence of anionic quenchers (Yaseen et al., 2014).

To examine the engagement amidst the Er complex and DNA, fluorescence quenching trials were conducted using KI as the quencher, both in the existence and lack of DNA (Figure 3A). The Stern-Volmer formula (Eq. 1) was applied to determine the suppressing coefficient (K_SV_). The computed K_SV_ values for the Er(III) compound by iodide ion, in the lack and existence of DNA, were 34.57 M^−1^ and 31.20 M^−1^, (as shown in Figure 3B). When KI solution was introduced in the existence of DNA, a distinct suppressing effect was seen in the Er(III)-DNA procedure. Notably, the suppressing intensity varied with increasing concentrations of KI. Consequently, the binding mode amidst the Er compound and DNA was identified as groove docking.

RETRACTED

**FIGURE 3:** **(A)** Fluorescence spectra of the Er-complex in the presence and the absence of KI and/or DNA. **(B)** The Stern–Volmer curves of the emission titration data.

#### 3.1.4 Comparative binding study

It is widely understood that the docking mode of Ethidium Bromide (EtBr) alongside DNA is through intercalation. EtBr is regularly utilized as a fluorescent explorer to verify the binding mode of DNA with tiny molecules (Jalali and Dorraji, 2017; Dong et al., 2018; Shi et al., 2018; Zhang et al., 2022a). In this study, the compound was included in a blend containing EtBr (8.0 × 10^−6^ M) and DNA (140 × 10^−6^ M), and the impact of the compound on the emission strength was computed. Upon intercalation into DNA, the fluorescence intensity of EtBr exhibits a significant increase. Similarly, if the compound interposes into DNA, it will reduce the available docking spots on DNA for EtBr. Consequently, this leads to a decrease in the emission strength of the DNA-EtBr compound. Figure 4A displays the fluorescence emission spectrum of the DNA-EtBr compound in the lack and existence of the Er compound. As depicted in Figure 4A, the DNA-EtBr compound exhibits a fluorescence emission maximum at 588 nm when excited at 525 nm. Interestingly, when the density of the Er compound is increased, the fluorescence strength of the DNA-EtBr compound only reduces by 10.4% (as shown in the inset of Figure 4A). This finding suggests that the docking of the Er compound with DNA differs from that of EtBr.

**FIGURE 4:** **(A)** Emission quenching curves of DNA-EtBr system by adding of Er complex. Inset is the plot of F/F_0_ vs. ([Complex]/[DNA]). **(B)** Effect of enhancing amounts of Er- complex on the DNA viscosity.

#### 3.1.5 Viscosity measurements

To delve deeper into understanding the engagement of the current Er- compound with DNA, researchers conducted viscosity experiments by altering the concentration of the complex introduced. The relationship between the comparative DNA viscosity (η/η_0_) and the comparative DNA length (L/L_0_) can be described using formula (L/L_0_) = (η/η_0_)^1/3^, where η_0_ and L_0_ represent the viscosity and the evident molecular range of DNA in the lack of the structure (Cheng et al., 2022).

Researchers performed viscosity experiments on a DNA solution with a concentration of 0.1 mM, while gradually adding more of the complex. The findings presented in Figure 4B show that there was no important alteration in the density of DNA alongside expanding amounts of the compound. Studying changes in DNA viscosity when a compound is added can provide insights into how the compound interacts with DNA. For compounds that intercalate amidst DNA bases, the DNA bases will separate to create space for the interposing molecule, causing an expansion in the relative DNA length and resulting in a higher DNA viscosity. In contrast, external interactions between compounds and DNA (such as docking to Significant or insignificant DNA grooves or through Coulombic forces) can farce the DNA helix to curve or spin, resulting in a small diminution in the effective DNA length and thus a diminish in DNA viscosity.

RETRACTED

#### 3.1.6 Effect of ionic intensity on the fluorescence properties

DNA, which contains phosphate groups, is a negatively charged polymer. To understand how small molecules interact with DNA, it is useful to monitor changes in the spectrum resulting from different levels of ionic strength. This method allows for investigating the impact of ionic strength and confirming the presence of electrostatic interactions. In this study, NaCl was employed to control the ionic strength of the solutions. The addition of Na^+^ ions increased the fluorescence strength of the molecule-DNA complex because of the contest for phosphate groups (Shahabadi et al., 2013). To assess this, the Er-complex was gradually exposed to NaCl in the lack and existence of DNA (4.4 μM), alongside NaCl densities ranging from (0–0.6 M). The outcomes revealed that the fluorescence strength of the compound-DNA mechanism and the liberated compound remained relatively unchanged, indicating that the docking amidst the Er compound and DNA was likely non-electrostatic.

### 3.2 Interaction with bovine serum albumin

#### 3.2.1 Fluorescence suppressing

Fluorescence Spectral analysis is a valuable procedure for obtaining valuable data about the interaction between a ligand and a protein (Nasir et al., 2017; Li et al., 2022; Wang et al., 2023). In Figure 5A, the fluorescence graph of BSA (3.0 µM) is displayed under various densities of the Er-complex (from 0 to 6.0 µM). The information demonstrates that the fluorescence strength of the BSA solution at 348 nm consistently decreases as the densities of the Er- complex increase. This indicates an engagement amidst BSA and the Er-complex, as the innate fluorescence of BSA is being quenched. Besides, there were no important shifts in the maximum emission wavelength of BSA, proposing that the Er-compound did not cause any noticeable configuration-based shifts in the compound of BSA. To analyze the emission strength information of BSA in the existence and lack of the Er-compound, the Stern-Volmer formula (Eq. 1) was employed (Sudha et al., 2016).

**FIGURE 5:** **(A)** Emission spectra of BSA in the presence and absence of different Er-complex amounts. **(B)** The F_0_/F vs. [Complex] curves at different temperatures.

RETRACTED

The K_SV_ numerical data representing the engagement between the stated compound and BSA were calculated for four different heat levels (295, 298, 300, and 303 K) by determining the incline of the linear plan of F_0_/F vs. [Q]. The results of these calculations are shown in Table 2 and visualized in Figure 5B. From the figure, it is obvious that the Stern-Volmer plans exhibit linearity, indicating the occurrence of just one model of suppressing procedure, static or dynamic. As exhibited in Table 2, K_SV_ decreases alongside expanding temperature. This suggests that the possible suppressing system for the docking of the Er compound to BSA is static.

**TABLE 2:** The Stern-Volmer constant (K_SV_), the binding constant (K_b_), number of the binding sites (n), and thermodynamic parameters (ΔS˚, ΔH˚, and ∆G˚) for the interaction of BSA with Er-complex at various temperatures.

(K) T	K_SV_ × 10^−5^ (M^−1^)	K_b_ × 10^−4^ (M^−1^)	n	ΔS˚ (J/mol.K)	ΔH˚ (kJ/mol)	∆G˚ (kJ/mol)
295	1.95 ± 0.03	7.76 ± 0.02	0.92			−27.61 ± 0.05
298	1.84 ± 0.03	5.89 ± 0.04	0.88	−216.33 ± 0.03	−91.53 ± 0.02	−27.21 ± 0.06
300	1.57 ± 0.06	4.26 ± 0.04	0.87			−26.59 ± 0.03
303	1.49 ± 0.02	2.95 ± 0.03	0.86			−25.92 ± 0.042

The calculation of the number of binding site (n) and K_b_ can be performed using Eq. 2 (Li et al., 2014). The linear equations for the temperatures 295, 298, 300, and 303 K are displayed in Figure 6A, and the matching computed factors are reported in Table 2. At 298 K, the binding constant (K_b_) for the Er compound was determined to be 5.89 × 10^4^ M^−1^, and the number of docking spots (n) was found to be close to 1. This shows a strong docking affinity amidst the Er compound and BSA, suggesting the formation of a unique binding site. This value of binding constant suggested that the binding of this complex with BSA is a non-intercalative interaction mode.

**FIGURE 6:** **(A)** The plot of log((F_0_-F)/F) vs. log([Complex]/µM) at four temperatures. **(B)** van’t Hoff plot for the interaction of Er- complex with BSA.

#### 3.2.2 Thermodynamic factors and nature of the docking forces

The incline and capture of a linear plan (Eq. 3) were utilized to determine the data of ΔH˚ and ΔS˚ built upon lnK_b_ vs. 1/T (also called the van’t Hoff Plot, as shown in Figure 6B. The thermodynamic factors for the engagement between the Er compound and BSA were compiled in Table 2. The fact that ΔG˚ was negative indicates that the docking of the Er compound to BSA is an unplanned procedure. Additionally, the negative numerical data of ΔH˚ and ΔS˚ indicate that hydrogen bonds and van der Waals engagement are the primary contributors to the binding between the Er compound and BSA.

RETRACTED

### 3.3 Docking procedure

#### 3.3.1 Docking study alongside DNA

To identify the optimal interaction site and conformation of the best compounds with the lowest energy on DNA, a docking study was conducted. The outcomes of the trial exhibited that the Er complex had the least docking energy and K_i_ for interacting with DNA at −6.8 kcal/mol and 16.43 μM (Table 3). As illustrated in Figure 7, the Er compound was positioned in the minor groove of the DNA. The binding free energy obtained from experimental and calculation results at 298 K for this complex is −24.93 and −28.42 kJ/mol, respectively. The existence of both non-polar and polar collectives in the Er compound facilitated its binding with DNA. Thus, based on both theoretical computer and trial procedures, it was concluded that the Er compound engaged with DNA via groove docking.

**TABLE 3:** The inhibition constants and binding energies of Er complex for the binding site of DNA and BSA.

Macromolecule	K_i_ (μM)	Binding energy (kcal.mol^−1^)
DNA	16.43	−6.8
BSA	9.46	−6.9

**FIGURE 7:** The docked model of the interaction between Er-complex and DNA.

#### 3.3.2 Docking study with BSA

The data presented in Table 3 indicates that site 3 exhibits the least docking energy of 6.91 kcal/mol, which aligns with the findings from the experimental techniques. Figure 8 shows that the Er compound is among specific amino acid remains, called LYS116, LYS136, GLU140, TYR137, TYR160, GLU125, LEU122, and ASP118. The binding free energy obtained from experimental and calculation results at 298 K for this complex is −27.21 and −28.84 kJ/mol, respectively. The presence of polar residues among these amino acids enables easy interaction between the complex and BSA via van der Waals forces and hydrogen bonding. The hydrogen bonding analysis in the molecular docking studies was performed and this study was observed without hydrogen bonding. Additionally, binding research conducted on other spots of BSA revealed that the Er compound exhibits a stronger docking effectiveness for site III (subdomain IB), which further supports the results obtained from the extermination studies.

**FIGURE 8:** The docked model of the interaction between Er-complex and BSA.

### 3.4 Anticancer analyze

The impact of the Er complex on HeLa and MCF-7 was investigated utilizing the MTT test. Figure 9 illustrates a graph depicting the percentage of cytotoxicity against varying concentrations of the Er complex. The results demonstrated that higher concentrations of the complex led to a reduction in the number of cancer cells. Within the concentration variety of 0.5–64 μg/mL, the Er complex exhibited toxicity of 18.1%–85.6% on MCF-7 cells and 17.2%–80.4% on HeLa cells. The IC_50_ values for the complex are provided in Table 4. It was observed that the maximum inhibition of cell growth occurred at a concentration of 100 μM.

RETRACTED

**FIGURE 9:** Plans of cytotoxicity percentage against the Er-complex concentrations against the MCF-7 and HeLa cell lines. Data are expressed as mean ± SD of three experiments.

**TABLE 4:** IC_50_ of this complex against the cell lines of HeLa, MCF-7 and human fibroblast cells (normal cells).

Cell lines	IC_50_ (µg/mL)
HeLa	7.01
MCF-7	7.54
Human Fibroblast	127.1

To assess the potential adverse effects of the Er-complex on non-cancerous cells, its cytotoxicity on human fibroblast cells was examined. Interestingly, the Er-complex demonstrated significantly lower cytotoxicity on non-cancerous human fibroblast cells compared to cancerous cells (Table 4). The highest mortality rate observed was 32.5% for fibroblast cells after 48 h of exposure to 100 μg mL^**−1**^ of the Er-complex, which was notably lower than the mortality rates observed for HeLa and MCF-7 cancer cells.

### 3.5 Antimicrobial action

The antimicrobial action of the compound was assessed, and it demonstrated promising results against the bacterial strains tested. Table 5 presents the antibacterial action of the Er compound vs. both $G^{+}$ and $G^{-}$ bacteria. The minimum inhibitory concentration (MIC) values ranged from 50 to 200 μmL^**−**1^. The findings suggest that this compound exhibited stronger antimicrobial impacts against *E. coli*.

**TABLE 5:** The antibacterial activity of Er-complex by the minimum inhibitory concentrations (MIC, µg/mL).

Bacteria or fungi	MIC (µg/mL)
P. aeruginosa	200
E. coli	50
E. faecalis	100
S. aureus	100

The antimicrobial capability of the compound can be ascribed to electron delocalization throughout the entire molecule, which expands its lipophilic character. This enhanced lipophilicity allows the complex to penetrate the lipid level of the microbial membrane more effectively, thereby preventing the metal docking spots on microbial enzymes. Chelation of the metal ion in metal compounds reduces its polarity, primarily because of the overlap of binding orbitals and partial sharing of the positive charge of the metal ion alongside the contributor clusters. Consequently, there is π-electron delocalization across the whole chelate ring, further enhancing the lipophilicity of the complex. While chelation is not the sole determinant of the complex’s antimicrobial activity, several other factors play a significant role. These factors include the dipole moment, size, geology of the complex, managing spots, electron transfer capability of the metal ion, dissolvability, bond length amidst the metal and binding, steric effects, density, and hydrophobicity. Taken together, these factors collectively contribute to the overall antimicrobial activity of the complex (Aramesh-Boroujeni et al., 2020).

RETRACTED

## 4 Conclusion

This analysis offers a comprehensive analysis of the docking of an Er compound with DNA and BSA in a physiological buffer. Various instrumental procedures were utilized to investigate the engagement system between the Er complex and DNA as well as BSA. The binding coefficient (K_b_), Stern-Volmer coefficient ( $K_{SV}$ ), and thermodynamic factors (ΔH˚, ΔS˚, and ΔG˚) were determined and documented. The fluorescence outcomes revealed that the Er compound interacts between DNA/BSA via a dynamic and static quenching procedure, respectively. The experimental findings propose that the Er compound binds to DNA through groove docking modes and interacts with BSA via hydrogen bonds and van der Waals forces. The outcomes from docking analysis indicate that the Er compound primarily binds to subdomain IB (site III) of BSA. Additionally, the antimicrobial and anticancer actions of the Er complex were assessed and found to be significant, demonstrating its strong antibacterial and anticancer properties. The findings of our current study provide valuable insights into the engagement mechanisms of tiny molecule compounds with DNA and BSA. This knowledge can be instrumental in further understanding the biological, pharmaceutical, and physiological implications of these interactions. Furthermore, the results obtained from this research hold potential for the development of future applications in these fields.

## Data Availability

The original contributions presented in the study are included in the article/Supplementary Material, further inquiries can be directed to the corresponding author.
